# Improving Image Quality and Reducing Scan Time for Synthetic MRI of Breast by Using Deep Learning Reconstruction

**DOI:** 10.1155/2022/3125426

**Published:** 2022-08-26

**Authors:** Jian Li, Lin-Hua Wu, Meng-Ying Xu, Jia-Liang Ren, Zhihao Li, Jin-Rui Liu, Ai Jun Wang, Bing Chen

**Affiliations:** ^1^Department of Radiology, General Hospital of Ningxia Medical University, Yinchuan, China; ^2^GE Healthcare China, Beijing, China; ^3^GE Healthcare China, Xi'an, China; ^4^School of Clinical Medicine, Ningxia Medical University, Yinchuan, China

## Abstract

**Objectives:**

To investigate a deep learning reconstruction algorithm to reduce the time of synthetic MRI (SynMRI) scanning on the breast and improve the image quality.

**Materials and Methods:**

A total of 192 healthy female volunteers (mean age: 48.1 years) underwent the breast MR examination at 3.0 T from September 2020 to June 2021. Standard SynMRI and fast SynMRI scans were collected simultaneously on the same volunteer. Deep learning technology with a generative adversarial network (GAN) was used to generate high-quality fast SynMRI images by end-to-end training. Peak signal-to-noise ratio (PSNR), mean squared error (MSE), and structural similarity index measure (SSIM) were used to compare the image quality of generated images from fast SynMRI by deep learning algorithms.

**Results:**

Fast SynMRI acquisition time is half of the standard SynMRI scan, and the generated images of the GAN model show that PSNR and SSIM are improved and MSE is reduced.

**Conclusion:**

The application of deep learning algorithms with GAN model in breast MAGiC MRI improves the image quality and reduces the scanning time.

## 1. Introduction

Magnetic resonance imaging (MRI) is essential for accurate diagnosis, staging, curative effect evaluation, and prognosis analysis of breast cancer. Conventional breast MRI includes T1WI, T2 STIR, DWI, and DCE-MRI images to comprehensively diagnose breast diseases. Quantitative magnetic resonance imaging is a new MRI technology that can obtain multiple tissue parameters (T1, T2, PD, R1, and R2) and multiple contrast images of the same sequence and level through one acquisition. Because of its unique advantages such as acquisition signal uniqueness, rapid synchronization, visualization, and multiparameter atlas, it has been gradually applied to the diagnosis of breast cancer, especially when T2 relaxation time has been proved to be an effective parameter for diagnosing breast cancer [1, 2]. However, the disadvantage of conventional breast quantitative MRI is long scanning time, which will reduce the tolerance of patients. At the same time, during long-time scanning, when patients appear to involuntarily move, it is easy to produce motion artifacts, which seriously reduces the image quality [3]. Synthetic magnetic resonance imaging (SynMRI) technology can be used to create any contrast weighted images, including T1-weighted, T2-weighted, and FLAIR images based on R1 and R2 relaxation rates (inverse ratio of T1 and T2 relaxation times) and proton density (PD). Due to the development of fast and synchronous relaxation measurement methods, SynMRI has become a clinically feasible method [4, 5]. These methods have high repeatability and reproducibility among different suppliers. However, even for SynMRI, the standard scanning still takes a long time. The scanning parameters can be adjusted to speed up the scanning, but the image quality will be lost. Therefore, reducing the simultaneous interpreting time of breast MAGiC MRI and developing a new technology that is equivalent to the quality of the traditional MAGiC MRI image are the key to solving this problem.

Deep learning technology with the generative adversarial network (GAN) is widely used to generate high-resolution images and improve image quality. The Generator and Discriminator are generated in competition and iteration, which are very close to the real image. A previous study points out that the GAN algorithm can improve the image quality of FLAIR MRI and effectively reduce its granularity [6]. Therefore, we hypothesize that GAN can generate high-quality fast SynMRI to shorten the scan interval to half to improve clinical efficiency.

## 2. Materials and Methods

### 2.1. Patients

This study obtained the permission of the ethics committee of the General Hospital of Ningxia Medical University and filled in the informed consent form for all the participants, and all data were fully anonymized before they were exported for research purposes.

From September 2020 to June 2021, the subjects who underwent breast MRI examination in the Department of Radiology of our hospital were selected as the subjects. According to the inclusion and exclusion criteria, 192 healthy volunteers were recruited. All subjects underwent routine breast MRI examination, standard SynMRI, and fast SynMRI scanning sequences. The inclusion and exclusion criteria are as follows.

Inclusion criteria are as follows: (1) healthy female volunteers who were recruited—all subjects who completed the routine breast MRI scans and breast SynMRI scans; (2) all subjects who were over 20 years old; and (3) non-postmenopausal patients who received magnetic MRI images of the breast in the second week of the menstrual cycle. Exclusion criteria are as follows: (1) those whose SynMRI images did not meet quality standards to be used as training targets of deep learning; (2) patients who are allergic to contrast agents, cardiac pacemakers, and claustrophobic patients who have terminated MRI scans; and (3) those with breast prosthesis, lactating, and pregnant women.

### 2.2. Image Quality Evaluation Criteria

MSE: mean squared error, a measure of the degree of difference between an estimated quantity and the actual quantity.

PSNR: peak signal-to-noise ratio, an objective criterion for evaluating images, which has limitations and is generally used as an engineering item between the maximum signal and background noise.

SSIM: the structural similarity index measure is a measure to evaluate the similarity between two digital images. Compared to traditional image quality measures such as peak signal-to-noise ratio (PSNR), the structural similarity index measure is a better measure of image quality than the human eye can judge [7].

### 2.3. MRI Scan Parameters

In this study, a 3.0 T magnetic resonance scanner (Signa Architect, GE Healthcare) and 8-channel phased array breast dedicated coils were used to scan patients and healthy volunteers. Volunteers were in the prone position with the feet advanced and the breasts on both sides naturally drooped and placed in the breast coil. The OAx SynMRI sequence is added to the routine clinical MR examination. The standard SynMRI scanning parameters are TR = 4000, 15000, TE = 9.4, 75.5, 84.9, 151, slice thickness 5 mm, spacing 0.5 mm, matrix = 320 × 256, FOV = 32 × 32, number of slices = 24, and the scan time is 5 minutes, 12 seconds. Our fast SynMRI scanning parameters are TR = 4000, 15000, TE = 9.2, 73.5, 82.7, 147, slice thickness 5 mm, spacing 0.5 mm, matrix = 320 × 256, FOV = 32 × 32, number of slices = 24, and the scan time is 1 minute, 52 seconds. Other scan parameters are shown in Table 1. Magnetic resonance image compilation (MAGiC) software was used to retrieve the quantification images T1, T2, and proton density (PD)—on the basis of the acquired data and to create synthetic T1-weighted (T1W) images, T2-weighted (T2W) images, and T2-weighted fluid-attenuated inversion recovery (T2W FLAIR) images [8].

### 2.4. Model Construction

In this section, due to decreasing the scan time of our SynMRI scan, we presented the SRGAN-based image clarity enhancement model, which makes scanning of images faster while ensuring clarity of images. Superresolution generative adversarial network (SRGAN) that we adopted from [9] is the network designed for estimating a high-resolution and superresolution image *I*^SR^ using a low-resolution image *I*^LR^ [10, 11]. *W* × *H* × *C* was described as tensor of size for image *I*^LR^ with *C* color channels, *rW* × *rH* × *rC* for *I*^SR^, respectively. As shown in Figure 1, unlike the regular generative adversarial network (GAN), SRGAN pioneered the introduction of GAN into the superresolution domain. The Generator's input in SRGAN is no longer noise, but *I*^LR^. And the structure of the Discriminator is no different from that of a normal GAN [11, 12]. We adopted [9] for the establishment and architecture of the SRGAN model due to its effectiveness in estimating high-resolution image *I*^HR^.

Involving GAN, we followed Goodfellow et al. [13] to define a Discriminator network *D*_*θ*_*D*__ along with Generator *G*_*θ*_*G*__ to solve the adversarial min–max problem:

(1) $$\begin{array}{c} \underset{\theta_{G}}{\min}\underset{\theta_{D}}{\max}E_{I^{\text{HR}}\sim p_{\text{train}}\left(I^{\text{HR}}\right)}\left[\log D_{\theta_{D}}\left(I^{\text{HR}}\right)\right]+E_{I^{\text{LR}}\sim p_{G}\left(I^{\text{LR}}\right)}\left[\log\left(1-D_{\theta_{D}}\left(G_{\theta_{G}}\left(I^{\text{LR}}\right)\right)\right)\right]. \end{array}$$

Generator contains three large modules between the input *I*^LR^ and the output *I*^SR^, as shown in Figure 2:

- A Conv layer with 3 × 3 kernels and 64 features plus a ReLU layer as the activation function
- B-residual blocks with identical layout proposed by Gross and Wilber [14], where each block contains two sets of Conv layers with 3 × 3 kernels and 64 features followed by Batch Normalization layer, plus a ReLU layer as the activation function. Each block uses the residual connection named Elementwise-Sum to add the block input to the block output, except the last block. An extra residual connection that added the input of first block to the output of last block was set for the Elementwise-Sum of last block
- Two Deconv layers and a Conv layer at last, each Deconv contains a Conv layer followed by two PixelShuffler layer, plus a ReLU layer as the activation function

The input of Discriminator is *I*^SR^ or *I*^HR^, and the output is the judgment results that tell if the input is a real image or an artificial image. Three modules contained between input and output are as follows:

- A Conv layer plus a Leaky ReLU as the activation function
- Seven blocks contained repeated Conv layer plus Leaky ReLU layer followed by BN layer. The size of kernel in each block increased periodically from 64 to 512, with the values of strides shifts cyclically between 2 and 1
- Dense fully connection layer plus Leaky ReLU layer as activation layer followed by Dense layer plus Sigmoid layer as activation layer at last. The role of fully connected layer is equivalent to adjusting the number of channels. The output of the last fully connected layer is (None, 32,32,1), which can be interpreted as 1024 discriminations, after which the 1024 results are aggregated to realize the discriminations of an image

### 2.5. Loss Function

The widely used loss function [15] is based on minimizing mean squared error to maximizing peak signal-to-noise ratio:

(2) $$\begin{array}{c} \text{MSE}=\frac{1}{H\times W}\overset{H}{\underset{i=1}{\sum }}\overset{W}{\underset{j=1}{\sum }}{\left(X\left(i,j\right)-Y\left(i,j\right)\right)}^{2}, \end{array}$$

(3) $$\begin{array}{c} \text{PSNR}=10\log_{10}\left(\frac{{\left(2^{n}-1\right)}^{2}}{\text{MSE}}\right). \end{array}$$

However, this common loss function is not applicable to GAN; the perceptual loss function *l*^SR^ adopted by [9] is critical for the performance of SRGAN. The authors formulated the loss function with a content loss and an adversarial loss component:

(4) $$\begin{array}{c} l^{\text{SR}}=l_{X}^{\text{SR}}+10^{-3}l_{\text{Gen}}^{\text{SR}}. \end{array}$$

*l*_*X*_^SR^ denotes the content loss and 10^−3^*l*_Gen_^SR^ denotes the adversarial loss.

#### 2.5.1. Content Loss

Content loss *l*_*X*_^SR^ on MSE is pixel-wised, calculated as

(5) $$\begin{array}{c} l_{\text{MSE}}^{\text{SR}}=\frac{1}{r^{2}WH}\overset{rW}{\underset{x=1}{\sum }}\overset{rH}{\underset{y=1}{\sum }}{\left(I_{x,y}^{\text{HR}}-G_{\theta_{G}}{\left(I^{\text{LR}}\right)}_{x,y}\right)}^{2}. \end{array}$$

This solution for maximizing PSNR often lacks high-frequency content to make images overly smooth. For general image, performance is still average; however, for MAGiC medical images such as near grayscale image, performance is below average.

Aiming for good performance on MAGiC image, VGG-19 feature extraction network [16] was introduced. To date, VGG-19 is still frequently used to extract image features [17]. VGG-19 requires only a small number of iterations to start converging and the network contains 16 Conv layers and 3 Full connection layers. The structure of VGG-19 is very consistent, using the 3 × 3 convolution and the 2 × 2 convergence from start to finish. The improvement of *l*_MSE_^SR^ is to define the VGG loss as the Euclidean distance between the feature representation of the artificial image *G*_*θ*_*G*__(*I*^LR^) and the real image *I*^HR^. This is done by feeding *I*^HR^ obtained from the Generator into the VGG network and calculating the Euclidean distance for each layer of the feature mapping:

(6) $$\begin{array}{c} l_{\text{VGG}/i,j}^{\text{SR}}=\frac{1}{W_{i,j}H_{i,j}}\overset{W_{i,j}}{\underset{x=1}{\sum }}\overset{H_{i,j}}{\underset{y=1}{\sum }}{\left(\phi_{i,j}{\left(I^{\text{HR}}\right)}_{x,y}-\phi_{i,j}{\left(G_{\theta_{G}}\left(I^{\text{LR}}\right)\right)}_{x,y}\right)}^{2}. \end{array}$$

*W*_*i*,*j*_ and *H*_*i*,*j*_ represent the dimensions of the respective feature inside the VGG network. *ϕ*_*i*,*j*_ is considered given to explicit the feature-map obtained by the *j*-th Conv before the *i*-th max-pooling layer in the VGG-19 network.

#### 2.5.2. Adversarial Loss

The loss function of GAN is based on the probability of the output of Generator. With adding GAN adversarial loss, the authors hope to confuse Discriminator on judging images produced by Generator:

(7) $$\begin{array}{c} l_{\text{Gen}}^{\text{SR}}=\overset{N}{\underset{n=1}{\sum }}-\log D_{\theta_{D}}\left(G_{\theta_{G}}\left(I^{\text{LR}}\right)\right). \end{array}$$

*D*_*θ*_*D*__(*G*_*θ*_*G*__(*I*^LR^)) represents the probability that *G*_*θ*_*G*__(*I*^LR^) was treated as *I*^HR^ by Discriminator.

### 2.6. Train Process

#### 2.6.1. Discriminator

Input the real image *I*^HR^ and the artificial image *G*_*θ*_*G*__(*I*^LR^) into the Discriminator. The loss is obtained from comparing the adjusting result of *I*^HR^ to 1 and *G*_*θ*_*G*__(*I*^LR^) to 0.

#### 2.6.2. Generator

**Step 1 .**

The artificial image *G*_*θ*_*G*__(*I*^LR^) is obtained by passing *I*^LR^ into Generator. The loss is obtained by comparing the discriminant result of *G*_*θ*_*G*__(*I*^LR^) with 1. This loss reflects whether the artificial picture generated by the Generator can deceive the Discriminator.

**Step 2 .**

Input the real image *I*^HR^ and the artificial image *G*_*θ*_*G*__(*I*^LR^) into the VGG feature extraction network to get the features of two images, and the loss is obtained by comparing the features of *G*_*θ*_*G*__(*I*^LR^) with those of real *I*^HR^. Notice: a new pair of *I*^LR^ and *I*^HR^ is needed for training process in Generator.

The model was implemented with PyTorch framework on Python platform (version: 3.6.8 https://www.python.org). Training and validation of our model were conducted on a local computing workstation, equipped with Intel Xeon CPU, NVIDIA Tesla V100 GPU, 64 GB of RAM. Training time by our SRGAN model was 19 hours.

### 2.7. Statistical Analysis

For quantitative evaluation, we calculated the mean squared error (MSE, equation (2)), peak signal-to-noise ratio (PSNR, equation (3)), and structural similarity index measure (SSIM, equation (8)) [15] for both numbers and images such as PD, T1, T2, T1W, and T2W. MSE in the image algorithm processes the mean value of the sum of squares of the difference between the image pixel value and the original pixel. PSNR is an objective standard for evaluating images based on MSE with a simple and fast algorithm. The PSNR shows how close the image reconstruction is to the source image on a logarithmic scale, and PSNR is one of the basic denoising metrics to validate the proposed algorithm. The evaluation metric SSIM analyzes the viewing distance, edge information between the reference and the test images, changed and preserved edges, textures, and structural similarity of the images. The range of SSIM is defined as 0 to 1. The more similar the two images are, the closer the value of SSIM is to 1. These calculation metrics can reflect the similarity of estimated high-resolution images and actual high-resolution images very effectively and accurately [15].

(8) $$\begin{array}{c} \text{SSIM}=\frac{\left(2\mu_{x}\mu_{y}+c_{1}\right)\left(\sigma_{xy}+c_{2}\right)}{\left(\mu_{x}^{2}+\mu_{y}^{2}+c_{1}\right)\left(\sigma_{x}^{2}+\sigma_{y}^{2}+c_{2}\right)}. \end{array}$$

*μ*_*x*_ is the average of *x*. *μ*_*y*_ is the average of *y*. *σ*_*x*_^2^ is the variance of *x*. *σ*_*y*_^2^ is the variance of *y*. *σ*_*xy*_ is the covariance of *x* and *y*. *c*_1_ = (*k*_1_*L*)^2^, *c*_2_ = (*k*_2_, *L*)^2^ are the constant used to maintain stability, which *k*_1_ = 0.01, *k*_2_ = 0.03, and *L* is the dynamic range of the pixel values, in general *L* = 255. Because not all the datasets were normally distributed when analyzed by the Shapiro-Wilk test, we used the nonparametric Wilcoxon signed rank test to compare the quantitative and qualitative scores. Two-way *P* value less than 0.05 was considered statistically significant. All the statistical analyses were performed using R (version: 4.1.0, https://www.rproject.org).

### 2.8. Ethics Statement

The study was conducted in accordance with the Declaration of Helsinki (as revised in 2013). This retrospective study was approved by the medical ethics committee of General Hospital of Ningxia Medical University (No. KYLL-2021-280), and written informed consent was waived due to the retrospective nature of the study.

## 3. Results

A total of 192 healthy volunteers were examined. The demographics of the study participants are summarized in Table 2. The three parameters previously mentioned (MSE, PSNR, and SSIM) of PDmap, T1map, T2map, T1W, T2W, and T2W Flair are shown in Table 3.

Figures 3–5 compare the results of GAN Fast MAGiC with those of regular MAGiC in terms of three quantitative parameters (PD, T1, and T2) and three weighted images (T1W, T2W, and T2W FLAIR), respectively, and the data for the generated images are obtained from the quantitative analysis of the table.

Our experimental data and the output images clearly show that the quality of our GAN Fast MAGiC MRI images is improved compared to that of the conventional MAGiC images, especially in T1W, T2W, and T2WFLAIR parameters. The PSNR metrics for T1W, T2W, and T2WFLAIR images improved from a median value of approximately 24 to 28, approximately 23 to 27, and approximately 24 to 27, respectively, and SSIM also improved approximately 0.1, 0.2, and 0.2, respectively. The improvement in both parameters indicates that GAN Fast MAGiC images have improved in visual error compared to the traditional MAGiC method and in comparing structural similarity consistent with Human Visual System (HVS) characteristics. Although the performance in quantitative parameters such as PD, T1, and T2 is the same as that of regular MAGiC, the improvement in weighted images can already show that the GAN Fast MAGiC model can output the same or even higher quality MRI images while reducing the scan time by half. A comparison of standard SynMRI and GAN images from the same patient is shown in Figure 6.

## 4. Discussion

The SynMRI technology scans to obtain the relaxation time of the tissue, and the quantitative information of proton density reflects the signal difference and pathological information of different tissues, which is of great significance for the identification of benign and malignant breast lesions. However, the disadvantage of SynMRI is that it takes a long time to scan in to obtain high-quality images and requires the patient to remain stationary for a long time, which is a challenging task for patients with breast cancer. Therefore, it is a great challenge to balance the scan time and image quality and the accuracy of the diagnosis.

For the moment, some clinical studies have applied deep learning technology to MRI of the head [18, 19] and abdomen [20], and these studies have yielded good results. According to research, the impact of GAN on image quality and its potential to reduce scan time in SynMRI of breast diseases has yet to be fully investigated. Our study compared standard SynMRI to fast SynMRI in a sample of bilateral breasts in healthy volunteers and showed that our experimental data and output images clearly demonstrated the improved quality of our GAN fast SynMRI images compared to standard SynMRI, especially in T1W, T2W, and T2WFLAIR images. The MRI scanning sequence, parameters, and scanning methods of healthy volunteers in this study were consistent with those of clinical breast cancer patients. So this result also applies to breast cancer patients. For patients with breast lesions, higher-quality SynMRI images can help to more accurately determine whether the tumor is benign or malignant. The metrics for T1W, T2W, and T2WFLAIR images improved from a median value of about 24 to 28, about 23 to 27, and about 24 to 27, respectively, and SSIM also improved by about 0.1, 0.2, and 0.2, respectively. The improvement in both parameters indicates that GAN Fast MAGiC images have improved in terms of visual error compared to the traditional MAGiC method and in terms of comparative structural similarity consistent with the Human Visual System (HVS). Although the performance in quantitative parameters such as PD, T1, and T2 is about the same as that of standard SynMRI, the improvement in weighted images can already indicate that the GAN model can output the same or even higher quality MRI images with half the scan time. The use of GAN algorithm in scanning SynMRI images of breast cancers is an innovative application of artificial intelligence, and our results proved that it has the potential to improve image quality, object detection accuracy, and radiologist confidence, as well as simultaneously reduce scan time to improve the patient tolerance of SynMRI examination on the breast. In conclusion, GAN algorithms can output the same or even higher quality MRI images with half the scan time of standard SynMRI, which facilitates the clinical application of SynMRI in the diagnosis of breast diseases and improves the efficiency of examinations.

This study has certain limitations: (1) the potential pathological and clinical conditions of the research subjects are different, and there is no comparison between conventional breast SynMRI images and deep learning reconstructed images for the actual diagnosis of breast diseases; and (2) it is a single-center, single-type research, which has certain limitations and lacks external verification.

## Figures and Tables

**Figure 1:** Discriminator and Generator training flowchart.

**Figure 2:** SRGAN network architecture diagram.

**Figure 3:** MSE of PD, T1, T2, T1W, T2W, and T2WFLAIR.

**Figure 4:** PSNR of PD, T1, T2, T1W, T2W, and T2WFLAIR.

**Figure 5:** SSIM of PD, T1, T2, T1W, T2W, and T2WFLAIR.

**Figure 6:** T1W, T2W, T2FLAIR, T1map, T2map, and PDmap images of standard SynMRI and GAN.

**Table 1:** Scan parameters.

Parameters	Ax T2 FLEX	Ax T1 FSE	Ax DWI b800	L-R Sag fs T2	Cor T2 FLEX	Standard SynMRI	Fast SynMRI
TR (ms)	4982	642	2517	5107	4292	4000, 15000	4000, 15000
TE (ms)	85	8	72	85	68	9.4, 75.5, 84.9, 151	9.2, 73.5, 82.7, 147
Slice thickness (mm)	5	5	5	4	4	5	5
Spacing (mm)	0.5	0.5	0.5	1	0.4	5	5
FOV	32 × 32	32 × 32	32 × 32	18 × 18	34 × 34	32 × 32	32 × 32
Number of slices	32	32	32	32	20	24	24
Scan time (min)	2	2	2	3.5	2	5	2

**Table 2:** Study population characteristics.

Variable	Result
Mean age (y)	48.1
Median age (y)	48
Mean diameter of mass (cm)	2.38 ± 1.61
Median diameter of mass (cm)	2.05

**Table 3:** Three parameters previously mentioned.

Variable	MSE	PSNR	SSIM
PD	102.989	23.714	0.772
T1	525112.632	15.557	0.631
T2	1231.180	15.160	0.599
T1W	32.630	24.858	0.810
T2W	13.174	26.240	0.869
T2W FLAIR	13.052	26.285	0.875

## Data Availability

The data used to support the findings of this study are available from the corresponding author upon request.
